# Effects of the Femoral Nerve Block and Adductor Canal Block on Tourniquet Response and Postoperative Analgesia in Total Knee Arthroplasty

This article has been retracted.

**DOI:** 10.1155/2022/2327753

**Published:** 2022-04-12

**Authors:** Di Jin, Yajuan Zhu, Fuhai Ji, Xiaoqi Kong

**Affiliations:** Department of Anesthesiology, First Affiliated Hospital of Soochow University, Jiangsu 215000, China

## Abstract

Tourniquet has emerged as an important role in surgical procedures, sixty patients undergoing elective total knee arthroplasty are randomly divided into the nerve block group and adductor duct block group in this paper. The changes of mean arterial pressure (MAP) and heart rate (HR) at different time points during operation, the changes of VAS scores at resting pain and exercise pain, and the changes of quadriceps femur muscle strength at different time points after operation are observed in 2 groups. The experimental results show that compared with adductor duct block, femoral nerve block can better relieve the intraoperative tourniquet reaction without affecting the postoperative analgesic effect and the muscle strength of quadriceps femurs.

## 1. Introduction

As a simple and practical method of hemostasis, tourniquet plays a very important role in surgical procedures, with the advantages of significantly reducing patient bleeding, providing the surgeon with a clear surgical field, and facilitating surgical operations [1–3]. Presently, it is commonly applied in total knee arthroplasty (TKA) [4]. However, the ischemic pain of the limb caused by the tourniquet also brings some pain and risk to the patient at the same time [5]. When the tourniquet has been used for a long period of time, patients may experience symptoms such as high blood pressure and increased heart beat rates. After the tourniquet is released, there are adverse reactions such as blood pressure drop or shock [6]. Therefore, it is often recommended for doctors to sedate patients with anesthesia, increase the dosage of opioids or other analgesics, or even add vasoactive drugs to alleviate such tourniquet reactions. In addition, for patients with coronary atherosclerosis and other cardiovascular diseases, the tourniquet reaction is more likely to cause myocardial ischemia and arrhythmia [7–9]. Similarly, radicals available in the limb ischemia can cause reperfusion injury which can also cause lung injury, which is not conducive to postoperative recovery of patients.

Simple nerve blocks are often used in anesthesia for lower extremity surgery, but the surgical site does not coincide with the tourniquet binding site and involves different nerves that are innervated by it [10, 11]. Studies shows that a lower limb nerve block can reduce tourniquet response, but the effect of various nerve blocks on tourniquet response is still inconclusive. Both the myocardial blockage and nerve blockage are common measures to control pain during and after TKA surgery.

The rest of this paper is organized as follows: Section 2 discusses related work and analysis, followed by the patient information and research methods in Section 3. Data statistics and comparative analysis are discussed in Section 4.  Section 5 concludes the paper with summary and future research directions.

## 2. Related Work

TKA is an effective surgical procedure for the treatment of advanced knee disease, but TKA often results in severe postoperative pain and impairs early functional exercise. However, TKA often leads to severe postoperative pain, which affects early functional exercise of the knee joint and increases the risk of postoperative complications such as knee stiffness and deep vein thrombosis, thus affecting the outcome of the surgery [12, 13]. Therefore, adequate postoperative analgesia after TKA is particularly important. The use of a single opioid analgesic dose is large and not ideal. Femoral nerve block and collecting duct block at the time of surgery can significantly reduce the amount of opioids used, which can obtain good analgesic effects and facilitate early postoperative movement of patients [14]. The adductor canal is located from the anterior superior iliac spine to the anterior medial aspect of the middle 1/3 of the patella, between the deep surface of the suture muscle, the greater trochanter and the medial femoral muscle. After the femoral nerve branches from the femoral triangle to innervate the quadriceps, it continues as a sensory branch of the saphenous nerve, which enters the collecting duct at the base of the femoral triangle and travels down the medial side of the knee after exiting the collecting duct and divides into the infrapatellar branch and the sutures muscle branch. The former is distributed on the anterior medial side of the knee joint, and the latter on the medial side of the calf and ankle [15]. When compared with femoral nerve blockage, the advantage of the adductor canal block does not affect quadriceps' muscle strength, which makes it to be a more preferred analgesic method.

The adductor canal is located from the anterior superior iliac spine to the anterior medial aspect of the middle 1/3 of the patella, between the deep surface of the suture muscle, the greater trochanter, and the medial femoral muscle. After the femoral nerve branches from the femoral triangle to innervate the quadriceps, it continues as a sensory branch of the saphenous nerve, which enters the collecting duct at the base of the femoral triangle and travels down the medial side of the knee after exiting the collecting duct and divides into the infrapatellar branch and the sutures muscle branch. The former is distributed on the anterior medial side of the knee joint and the latter on the medial side of the calf and ankle [16].

The current tourniquet reaction can be considered as a systemic reaction which is caused by the ischemia-reperfusion injury as a result of the tourniquet compression of local tissues and the transmission of the injury signal through the local peripheral nerves. The results of this study show that the MAP change in the femoral nerve block group has a higher stability rate as compared to that of the adductor tube block group. This may be due to the fact that the effect of the adductor tube block is lower than the tourniquet binding site, so the compression effect of the tourniquet cannot be relieved. The femoral nerve block can more effectively block the upward conduction of stimulation there, thereby alleviating the tourniquet response. In addition, there is still a difference in MAP between the femoral nerve block group and the adductor tube block group. There is a corresponding change in MAP with the change of the tourniquet time, indicating that the femoral nerve block or the adductor muscle alone cannot completely eliminate the influence of tourniquet reaction. Studies shows that even with sufficient sensory levels in spinal cord and epidural anesthesia, tourniquet pain and high blood pressure will also occur, and the peripheral nerve block has not been proven to be completely effective in preventing blood bands [17, 18]. Therefore, the mechanism of tourniquet reaction remains to be further studied.

Patients with TKA need to start rehabilitation exercises and get out of bed as soon as possible after surgery in order to facilitate their knee function recovery. However, 50% to 60% of patients have severe postoperative pain that interferes with early postoperative functional exercise, which in turn affects the functional recovery of the knee and also increases the risk of deep vein thrombosis and pulmonary embolism. The pain is mainly due to muscle ischemia-reperfusion injury which is caused by quadriceps spasm, intraoperative tourniquet binding, and release of inflammatory mediators. Therefore, effective analgesic treatment after TKA is essential for the recovery of knee function.

## 3. Patient Information and Research Methods

### 3.1. Patients and Treatment

Clinical trials are performed on patients undergoing knee arthroplasty who are admitted to the Department of Orthopedic Surgery in the First Affiliated Hospital of Suzhou University from July 2020 to March 2021.

1. Entry criteria: The American Society of Anesthesiologists (ASA) created two groups, grade I∼II, and age 51–80 years old. In the end, about 60 cases are included, and they are randomly divided into the femoral nerve block group and the adductor carnal block group by the random number table method, with 30 cases in each group. There is no statistically significant difference between the two groups of patients in general data such as gender, age, BMI index, and length of operation (*P* > 0.05), and they are comparable, as shown in Table 1.
2. Exclusion criteria: there are some patients who refuse to participate in this trial, these patients either have medical-related problems such as cognitive dysfunction, poor communication, peripheral neuropathy or potential peripheral neuropathy, local skin infection, clotting dysfunction, drug allergy, and drug addiction. Table 1 shows the comparison of the femoral nerve block group and adductor tube block group.

All patients did not use preoperative medication before entering the room. After a patient enters the room, the peripheral vein is opened, and the monitor is connected to monitor blood oxygen saturation, electrocardiogram, non-invasive blood pressure, and the radial artery puncture method is used to monitor the invasive arterial blood pressure. The patients were administered general anesthesia with endotracheal intubation. The patients are pumped with dexmedetomidine 0.5 *µ*g/kg for 10 minutes before induction. Propofol 1.5–2 mg/kg, sufentanil 0.4–0.6 *µ*g/kg, and cis-atracuron besylate were used at 0.15–0.2 mg/kg for anesthesia induction, sevoflurane inhalation. Anesthesia is maintained by intermittent bolus injection with cis-benzene, and the depth of anesthesia is monitored by inhalation anesthetic concentration monitoring (MAC0.8-1.2Vol%).

After induction, B-ultrasound (Wisonic Huasheng, model: Navi S) guides the nerve block. The patients in the femoral nerve block group are placed in a supine position, and a high-frequency ultrasound probe is placed along the horizontal axis near the groin of the lower extremity on the operating side. The femoral nerve is located outside the femoral artery. The needle is inserted into the outside of the thigh by the in-plane method, and the needle tip reached around the femoral nerve. After confirming that the blood vessel is not inserted, 20 ml of 0.2% ropivacaine is injected. In the adductor tube block group, the inferior sartorius approach is often used. The patient's affected limb is slightly externally rotated. The ultrasound high-frequency probe is placed horizontally on the middle of the thigh on the operating side to confirm the position of the sartorius muscle. 20 ml of 0.2% ropivacaine is injected. The space between the sartorius muscle and its fascia and the artery.

### 3.2. Observable Indicators

#### 3.2.1. Intraoperative Hemodynamic Changes May Occur in Two Groups of Total Knee Arthroplasty Patients

  Observing the intraoperative steps: *T*0 means before anesthesia, *T*1 means upper tourniquet immediately, *T*2 means upper tourniquet for 30 min, and *T*3 means upper tourniquet for 60 min.
  The changes of mean arterial pressure MAP and heart rate HR in patients with:*T*4 means 90 minutes from the upper tourniquet, *T*5 means the tourniquet is loosened, and *T*6 means 10 minutes after the tourniquet is loosened.

#### 3.2.2. Postoperative Pain of the Two Groups of Total Knee Arthroplasty Patients

The resting VAS (visual analog scale) score and exercise VAS score of patients at 6 h and 24 h after operation was observed. 0 is painless, (1–3) is mild pain, (4–7) is moderate pain, and (8–10) is severe pain.

#### 3.2.3. Quadriceps Muscle Strength of the Two Groups of Patients Undergoing Total Knee Arthroplasty

It was observed that the quadriceps muscle strength of the patients are affected limb at 6h and 24h after surgery that no muscle contraction at all is level 0. Only muscle contraction cannot. The resulting movement is level 1. The affected limb can move in the horizontal direction but cannot resist gravity is level 2. It can be lifted off the bed surface but cannot resist resistance is level 3. The resistance that can resist is not completely level 4, and the muscle strength is normal level 5.

### 3.3. Statistical Processing

The research uses data collection packages such EXCEL2016 and SPSS23.0 for research data analysis. The measurement data in the research data all pass the normality test and are described by the mean *X* ± SD. The comparison between the two groups is the group *t*-test or the adjusted Test (statistic is T), and the before and after comparison within the group is the paired *t*-test (statistic is t). Repeated measurement analysis of variance (statistics is F) + LSD-t test for comparison between two groups (statistics is LSD-t) + pairwise time comparison difference *t* test (statistics is t). The count data are described by the number of cases, and the comparison between the two groups is the chi-square test or the adjusted chi-square test (the statistic is *χ*^2^). The statistical test level *α* = 0.05, both are two-sided tests. The multiple comparisons of repeated measurement analysis and segmentation test are adjusted according to the Bonferroni correction method, *α*′ = 0.05/*n*, *n* is the number of multiple comparisons.

## 4. Data Statistics and Comparative Analysis

### 4.1. Changes in Mean Arterial Pressure (MAP) at Different Time Points in the Two Groups of Patients

The mean arterial pressure MAP data and data of the two groups of patients at different time points during the operation are listed in the table below. The overall comparison (two-factor repeated measurement variance) shows that between groups (grouping latitude), within groups (time latitude), and interaction (between groups × time), all have a significant significance (*P* < 0.05). Two-by-two fine comparison combined with main data analysis: there is no statistically significant difference in basic MAP between the two groups (*P* > 0.05). The upper tourniquet immediately, 30 min, 60 min, 90 min, the tourniquet immediately, and 10 min at each time point of the two groups of patients The difference in MAP is statistically significant (*P* < 0.05). The MAP during the upper tourniquet in the femoral nerve block group is lower than that in the adductor tube block group. After the tourniquet is released, the MAP is higher than that in the adductor tube block group. In comparison within the group, with the extension of the tourniquet time, the MAP is increased. After the tourniquet is released, the MAP is decreased, which is significantly different from the *T*_0_ time point (*P* < 0.008, *X*±SD, *n* = 30), as shown in Table 2.

The overall comparison is a two-factor repeated measurement analysis of variance. The fine comparison between groups in latitude is LSD-t test, and the significance markers and *b* are *P* < 0.05 compared with groups A and B, respectively. The fine comparison in time latitude is the difference *t*-test, and the significance mark *t* is *PP*<*α*′ compared with the first time point in the group. *α*′ = 0.05/6 = 0.008, 6 is the number of multiple comparisons (Bonferroni correction method).

### 4.2. Changes of HR in the Two Groups of Knee Patients at Different Times during the Operation

The overall comparison of the simulation upward shows that only within the group (time latitude) has a significant meaning (*P* < 0.05). Two-by-two fine comparison combined with main data analysis: there is no statistically significant difference in heart rate at each time point between the two groups of patients (*P* > 0.05); within each group, there is no change in the snack rate of patients in the femoral nerve block group at each time significant difference (*P* > 0.05), the difference of HR over time in the adductor tube block group (compared with *T*0) is statistically significant (*P* < 0.008), as shown in Table 3.

### 4.3. VAS Pain Score and Quadriceps Muscle Strength Changes in the Two Groups of Patients at Different Time Points after Surgery

There is no statistically significant difference in the VAS scores of resting pain between the two groups of patients at 6 h and 24 h after surgery (*P* > 0.05), and there is no significant difference in the VAS scores of exercise pain between the two groups at 6 h and 24 h after surgery (*P* > 0.05). There is no statistically significant difference in quadriceps muscle strength between the group of patients at 6 h and 24 h after surgery (*P* > 0.05). However, the sport VAS score and quadriceps muscle strength of the femoral nerve block group at 24 hours after operation are significantly changed. Compared with 6 hours after operation, the difference is statistically significant.  Table 4 shows the pain scores and quadriceps muscle strength of the two groups of patients 6 hours after surgery.

### 4.4. Comparison of Sports VAS Scores and Resting VAS Scores in Each Group

The sports VAS scores of each group are higher than the resting VAS scores, and the difference is statistically significant (*P* < 0.05), as shown in Table 5.

## 5. Conclusions

This article intends to comprehensively compare the effects of two nerve block methods on tourniquet response and postoperative analgesia and explore a more favorable nerve block method for TKA patients. There is no significant difference in intraoperative HR changes between the femoral nerve block group and the adductor tube block group, and both are relatively stable, which may be related to the use of dexmedetomidine. Studies show that tourniquet reaction is related to increased sympathetic tone, so the antisympathetic effect of dexamethasone can help alleviate tourniquet reaction. Comparing the two groups, there is no significant change in HR in the femoral nerve block group, and there are statistical differences in HR changes in the adductor tube block group, indicating that the femoral nerve block group could better control the increase in heart rate caused by the tourniquet reaction.

Presently, the adductor tube block is more used for postoperative analgesia after TKA, and the main consideration is that the femoral nerve block will cause the decrease of quadriceps muscle strength and affect postoperative recovery. Theoretically, low concentrations of ropivacaine have little effect on the muscle strength of the blocked area, but studies show that ropivacaine can achieve sufficient analgesic effects within the concentration range of 0.1%–0.2%, so it with 0.2% ropivacaine for femoral nerve block, there is no significant difference in the analgesic effect and quadriceps muscle strength between the two groups of patients after surgery, which is consistent with the results of the previous study. Therefore, the use of low-concentration ropivacaine for femoral nerve block has no significant decrease in quadriceps muscle strength compared with adductor tube block, and it will not affect the early functional exercise of patients after knee arthroplasty.

## Figures and Tables

**Table 1:** Comparison of the two groups of patients.

*n*		Age	Height (cm)	Weight (kg)	BMI (kg/m^2^)	Operation time (h)	Sex ratio (M : F)	ASA group index I/II
Femoral nerve block group	30	66.37 ± 10.70	158.93 ± 6.59	68.67 ± 10.98	27.15 ± 3.61	2.89 ± 0.90	7/23	10/20
Adductor tube block group	30	68.40 ± 6.84	160.50 ± 7.07	68.40 ± 12.43	26.49 ± 4.17	2.90 ± 0.88	8/22	7/23
*t* (*χ*^2^)		0.876	0.890	0.089	0.655	0.044	0.089	(0.739)
*P*		0.386	0.377	0.929	0.515	0.965	0.766	0.390

**Table 2:** Mean arterial pressure MAP (mmHg) changes at different time points in the two groups of patients during operation.

	Femoral nerve block group	Adductor tube block group
*T*0	107.878 ± 11.904	108.573 ± 16.352
*T*1	91.287 ± 8.516*t*	98.918 ± 13.423*at*
*T*2	88.490 ± 10.571*t*	96.924 ± 12.668*at*
*T*3	91.389 ± 13.203*t*	102.555 ± 9.743*a*
*T*4	93.785 ± 12.603*t*	106.302 ± 10.069*a*
*T*5	87.672 ± 13.444*t*	75.638 ± 10.565*at*
*T*6	85.000 ± 13.329*t*	73.539 ± 10.826*at*

HF factor is given as 0.9833, *P* is 5.378 of groups F, *P* is 40.686 of F in the group, and *P* is 10.644 of correlations.

**Table 3:** HR changes at different time points during the operation of the two groups of patients (bpm).

	Femoral nerve block group	Adductor tube block group
*T*0	71.965 ± 11.755	72.580 ± 8.940
*T*1	59.169 ± 8.534*t*	59.614 ± 8.133*t*
*T*2	59.440 ± 10.254*t*	60.708 ± 9.314*t*
*T*3	63.061 ± 12.079*t*	63.464 ± 11.201*t*
*T*4	65.996 ± 11.916*t*	65.030 ± 8.646*t*
*T*5	66.154 ± 11.162*t*	67.748 ± 11.779*t*
*T*6	65.086 ± 10.470*t*	68.498 ± 9.541*t*

HF coefficient is given as 0.9601, *P* is 0.763 of groups F, *P* is 11.468 of F in the group, and *P* is 0.263 of correlations.

**Table 4:** Pain scores and quadriceps muscle strength of the two groups of patients 6 hours after surgery.

		Resting VAS score	Exercise VAS score	Quadriceps muscle strength
Femoral nerve block group *n* = 30	Postoperative 6 h	1.63 ± 0.56	2.40 ± 0.56	2.80 ± 0.76
	Postoperative 24 h	1.40 ± 0.56	1.97 ± 0.62	3.53 ± 0.51
	Difference	−0.23 ± 1.21	−0.43 ± 0.47	0.73 ± 0.21
	Paired test, *P*	1.041, 0.306	5.011, <0.001	19.040, <0.001
Adductor tube block group *n* = 30	Postoperative 6 h	1.60 ± 0.62	2.20 ± 0.81	2.77 ± 0.68
	Postoperative 24 h	1.38 ± 0.57	2.13 ± 0.78	3.57 ± 0.50
	Difference	−0.22 ± 0.94	−0.07 ± 1.72	0.80 ± 1.13
	Paired test *t*, *P*	1.282, 0.210	0.223, 0.825	3.878, 0.001
Comparison	Postoperative 6 h	0.197, 0.845	1.112, 0.271	0.161, 0.873
(Group test *t*, *P*)	Postoperative 24 h	0.137, 0.892	0.880, 0.382	0.307, 0.760

**Table 5:** Comparison of sports VAS scores and resting VAS scores in each group.

		Resting VAS score	Exercise VAS score	*t*	*P*
Femoral nerve block group	Postoperative 6 h	1.63 ± 0.56	2.40 ± 0.56	5.325	<0.001
*n* = 30	Postoperative 24 h	1.40 ± 0.56	1.97 ± 0.62	3.737	<0.001
Adductor tube block group	Postoperative 6 h	1.60 ± 0.62	2.20 ± 0.81	3.222	0.002
*n* = 30	Postoperative 24 h	1.38 ± 0.57	2.13 ± 0.78	4.252	<0.01

## Data Availability

Data from simulated experiments used to support the findings of this study are available from the corresponding author on reasonable request.
